RETRACTED

# Yolo-Based Traffic Sign Recognition Algorithm

**DOI:** 10.1155/2022/2682921

**Published:** 2022-08-03

**Authors:** Ming Li, Li Zhang, Linlin Li, Wenlong Song

**Affiliations:** ^1^College of Information and Computer Engineering, Northeast Forestry University, Harbin 150040, China; ^2^Cai Ji Center Primary School, Suqian 223813, Jiangsu, China; ^3^Northeast Forestry University, Harbin 150040, China

## Abstract

With the rapid development of intelligent transportation, more and more vehicles are equipped with intelligent traffic sign recognition systems, which can reduce the potential safety hazards caused by human cognitive errors. Therefore, a more safe and reliable traffic sign recognition system is the demand of drivers, and it is also the research hotspot of current automobile manufacturers. However, the pictures taken by the actual driving car are inevitably distorted and blurred. In addition, there are external uncontrollable factors, such as the impact of bad weather, which make the research of traffic sign recognition system face many difficulties, and the practical application is far from mature. In order to solve the above challenges, this paper proposes a Yolo model for traffic sign recognition. Firstly, the traffic signs are roughly divided into several categories and then preprocessed according to the characteristics of various types of signs. The processed pictures are input into the optimized convolutional neural network to subdivide the categories to obtain the specific categories. Finally, the proposed recognition algorithm is tested with the data set based on the German traffic sign recognition standard and compared with other baseline algorithms. The results show that the algorithm greatly improves the running speed on the basis of ensuring a high classification accuracy and is more suitable for traffic sign recognition system.

## 1. Introduction

With the rapid development of economy and the rapid progress of science and technology, the vigorous development of the automobile industry has gradually made cars enter most families, bringing people infinite convenience and many negative effects. As the growth rate of vehicles is much higher than the speed of road construction, people travel, and material exchanges are frequent, road traffic congestion and safety problems are becoming more and more serious. At the same time, the environmental problems brought about by it have become increasingly prominent, especially endangering the urban environment. Automobile exhaust and other system diseases have caused high ozone content in the surface air, aggravating the urban heat island effect. Light pollution is also a major problem of modern urban pollution. The rapid development of intelligent transportation system provides powerful technical application support for solving this kind of problems. It effectively applies science and technology such as information technology, data communication technology, sensor technology, and artificial intelligence to transportation, service control, and vehicle manufacturing. It is an integrated transportation management system. Intelligent transportation system has become an internationally recognized fundamental way to solve general traffic problems and has been paid more and more attention and widely used by governments, experts, and scholars at home and abroad. Intelligent transportation system has developed from the intellectualization of a single transportation element to the integration of transportation elements.

RETRACTED

As a part of intelligent transportation system, TSR system has become one of the research hotspots of scholars at home and abroad. The main task of the identification system is to ensure that the identification information is transmitted to the driver timely and effectively through the detection and identification of traffic signs, so as to reduce traffic congestion and ensure traffic safety. Road traffic signs are composed of different characters and patterns, and have different colors and shapes. When the TSR system is driving, the data acquisition equipment at the front end processes the collected traffic sign images into digital signals, which are used as the input of the signal processing system. After detection, classification, and recognition by the operation control system, the recognition results are output to the back-end alarm system. It is suggested that the driver should take countermeasures such as emergency braking or sign maintenance notice.

On the one hand, the driver should be warned in time to ensure smooth traffic and prevent accidents. On the other hand, driverless driving is a hot research topic in the field of advanced driving technology at this stage. In this research, TSR is an important part. It can directly control the vehicle by replacing the driver to ensure that the embedded and real-time information collection can transmit some important road traffic signals to the driverless system. Therefore, an efficient, real-time, and accurate TSR system is one of the important performances of future driverless vehicles.

## 2. Related Work

In the 1970s and 1980s, many countries have explored the road traffic sign recognition system. However, in view of the limitations of information technology at that time, mainly the limitations of computer computing performance, some technologies did not make great breakthroughs. In recent years, automobile manufacturers in various countries have paid more and more attention to this skill, and commercial products have emerged accordingly. For example, the traffic sign recognition system applied to BMW 7 series is based on the cooperation between Mobileye and continental. Subsequently, Mercedes-Benz S-class series cars were further improved. The front camera and special processor were combined to identify the speed limit signs. In addition, on the basis of traditional identification, dynamic LED identification is also supported. Subsequently, the types of identified traffic signs have been continuously increased and have been applied in Volkswagen Phaeton series and Volvo series cars. Although the above commercial applications have achieved some success, the types of recognition are few after all, and the spatial range of detection is also very limited.

RETRACTED

The algorithm of traffic sign recognition system mainly includes the following modules: image restoration (preprocessing), sign detection, and sign classification and recognition. According to different stages of processing, before detection, the degraded image should be inversely transformed to get a relatively clear image. Detection is to locate the Rio that may contain traffic signs from the natural environment and input the detection results into the classification and recognition stage. Identification classification and recognition is to use different methods to extract the features of the above areas that may contain traffic signs, and classify the areas of interest through appropriate classification algorithms to obtain the classification categories of traffic signs, and then subdivide them to obtain specific categories. Due to the influence of rain, snow, haze, sand and dust, and other bad weather on the image, it is mainly manifested as occlusion and contrast reduction. In fact, it is equivalent to adding interference. Simple filtering or color enhancement can be applied to the image to better restore the image. However, these complex and changeable backgrounds in reality will greatly affect the detection and recognition effect of the system.

### 2.1. Research Status of Traffic Sign Detection

The image detection technology used at this stage has already replaced the manual investigation method and is developing toward a more and more intelligent direction. In traditional image detection, it is necessary to avoid missed detection and false detection, because the classification and recognition in the later stage is the region of interest for processing the detection output. If false detection occurs in the detection stage, it will lead to the false detection of the entire system in this identification. When applied to auxiliary driving and intelligent vehicles, high real-time performance should be considered. In view of the outdoor environment of traffic signs, the detection phase faces some practical problems, such as lighting conditions. As the two most significant and stable features of traffic signs, color and shape have attracted more and more attention, and many different targeted detection methods have been designed by using this feature.

RETRACTED

#### 2.1.1. Color-Based Threshold Segmentation

The color-based traffic sign detection algorithm first intercepts the points of a specific color from the pattern and then filters the regional features after connecting them into regions, that is, constructs the mathematical model of color regions to output the regions of interest that may contain traffic signs. RGB color mode is one of the most widely used color systems at present, namely, red, green, and blue. Other colors are composed of the components of these three colors according to a certain proportion. Generally, images can be represented by RGB three primary colors. The segmentation method based on RGB [1–5] threshold is to set an interval range for red, yellow, and blue, respectively, according to the red, yellow, and blue primary colors of traffic signs. The threshold range is obtained by experiments, and then all pixels in the image are divided according to this threshold. This algorithm has fast processing speed and is not easy to be affected by visual angle. Reference [6] proposed a color image segmentation method based on RGB spatial color similarity. It is based on color information and brightness information, combined with the proposed image color component calculation method to form a color classification map. Finally, pixel segmentation is carried out according to the color classification map. This method not only ensures low complexity, but also improves accuracy. Literature [7–9] proposes an algorithm that effectively combines the depth learning technology and RGB image features, and uses the characteristics of the depth learning model to improve the accuracy of object recognition. Because the image color is easily affected by illumination, the difficulty of the algorithm depends on how to adapt to different illuminations in the process of color extraction. Janssen et al. divided the three components of RGB by the three components, respectively, and normalized the RGB components.

The above algorithm is limited to different lighting conditions and may be missed. Some scholars have converted RGB color space to his space [10]. *H*, *I*, and *s* in his [11–14] space are expressed as hue, color saturation, and brightness, respectively, and the three components are independent. Hue and chroma can eliminate the influence of lighting, but the amount of calculation is large, which is not conducive to the scene with high real-time performance. Literature [15] designed YUV space and his space conversion algorithms, which greatly improved the speed and accuracy of real-time video image processing. In addition, lab [16], YCB cr [17], and LUV [18] spaces can be used for conversion, but they are not widely used in general.

RETRACTED

Gomez-Moreno et al. [19] summarized the recognition effects in various color spaces. The results showed that in a complete set of traffic sign detection and classification system, the detection results of normalized RGB space and HSV space were better than other color spaces, and the two were similar. In addition, researchers combine the points with the same color and close location as the region of interest. This color lookup technology can detect the recognition efficiency as soon as possible, and there is a corresponding color lookup table. Escalera et al. combined with corner detection to find the region of interest, but this method cannot solve the problem caused by occlusion in the binary image composed of adjacent color points. Region growth uses the adjacent color points to connect the adjacent color points into a series of connected regions. Because the connected regions contain some false alarms, if they are directly output as regions of interest, it will bring a great burden to the subsequent classification work. By judging the size and aspect ratio of each connected region, some false alarms can be quickly eliminated.

Some simple criteria such as size and aspect ratio are only a method to quickly eliminate some simple false alarms. There will still be a large number of false alarms in the filtered image. Therefore, the improved algorithm further filters by judging the shape of the connected domain. Maldonado-bascón [20] et al. proposed the distance to the feature of the bounding box. The proposed method, combined with linear support vector machine, can cover the distance between the four edges of its smallest rectangle. Researchers calculate the shape based on this distance and construct feature vectors from the points in the shape. Then, the support vector machine (SVM) recognizes the feature vector. If the recognition result is not the shape of the traffic sign, it will be screened out; Jia et al. [21] calculated the distance from the center of the connected domain to all its edges and described it as a one-dimensional curve. Finally, after calculating the FFT amplitude feature, input the nearest neighborhood classification or neural network classifier to judge the shape [22–24]. The results show that this method has good invariance to translation and rotation, but the disadvantage is that the algorithm is expensive; other scholars use the features of the tangent function to construct the feature vector Xu [25]. First, they calculate the tangent angle of each point of the edge curve of the connected region formed by region growth, use the tangent value of the tangent angle to construct the feature vector, and complete the classification through template matching. The above algorithms mainly use the feature extraction based on color features. Although other methods can be used to enhance the reliability in the process of color extraction, it cannot avoid special conditions. When there are multiple identifications connected together, or the background color is fuzzy and difficult to distinguish in time, it is difficult to extract the connected domain. Lack of light or serious fading of signs will also occur, which will cause the color-based method to be unstable or even miss detection, and the detection accuracy will be reduced. At this point, shape-based detection algorithm can better solve these problems.

RETRACTED

#### 2.1.2. Shape-Based Traffic Sign Detection and Feature Extraction

Shape feature is an important visual feature of image, which is as stable as color feature. The corresponding detection technology first extracts features from the image shape and then detects. There are two commonly used representation methods for shape features: one is contour feature, and the other is region feature. The contour feature mainly refers to the external edge of the image, while the regional feature of the image refers to the whole shape of the image. Among the methods for describing the boundary features of images, the early method is template matching method, which uses the principle of template matching pixel by pixel in the image [26]. According to the experiment, a threshold is determined. The region with the lowest matching cost is the target region to be detected. The typical algorithms are Haar [27] and the method based on square gradient histogram (HOG) [28]. Some studies have extracted Haar features in specific color channels to detect traffic signs and achieved good results [27, 29, 30]. Taking advantage of the strong discrimination of gradient histogram, it is used as a shape descriptor to cooperate with SVM to achieve high accuracy.

Hough [31] transform, as a commonly used shape detection method, uses the principle of point line duality to form a closed boundary of pixels connecting the edge. A histogram is made according to the size and direction of the edge after the edge of the image is located by the differential calculation method. The disadvantage is that the computation cost of transformation is large and the storage space is high. Some scholars have improved the Hough transform algorithm, which greatly reduces the amount of computation. Loy and Zelinsky [32] proposed a diameter symmetry algorithm based on Hough transform, one of which is to calculate the gradient direction of edge points according to the symmetry law of circular diameter; Ruta [33] combines color feature information to greatly improve the efficiency of the algorithm. Loy and Barnes [34, 35] expanded the application field on this basis and applied the mirror symmetry algorithm to triangle and square identification detection, but the detection accuracy is not as high as that of the circle, and there is also a gap in real-time performance. Later, Belaroussi and Tarel [36] improved the Hough algorithm on triangle identification, and the real-time performance was improved. In general, Hough transform based on shape features can solve the occlusion problem to a certain extent, but the types of traffic sign shapes detected are limited; especially when the image is deformed due to angle tilt, the efficiency is significantly reduced.

RETRACTED

When geometric parameters [37] are actually applied to shape expression and matching, it is simpler to use them as feature descriptions. For example, the shape parameter method using the quantitative measure of related rectangles as parameters is a regional feature description method. In addition, there is a shape invariant matrix, which uses the moment of the region occupied by the target as the parameter of shape description. Some methods can also effectively detect shape features by combining with genetic algorithm. Tibaijuka et al. [38] first used Laplace kernel filter to capture the region of interest from the image and convert it into a binary image. Then, the genetic algorithm is used to search and detect the target shape. In the traffic sign detection, the genetic algorithm can effectively adapt to the sign deformation. However, the disadvantages are also obvious; that is, only one can be detected at a time, and multiple calls are required when detecting multiple identifiers at the same time, which means that genetic algorithm is not suitable for high real-time environment. In recent years, it has studied the advantages of integrated shape and color. On the problem of traffic sign detection, it has proposed a method of combining color information with shape features. Color segmentation is carried out first. On this basis, the method of shape feature analysis is used for recognition, and the effect is good. In general, whether it is color-based traffic sign detection, and shape-based or template matching-based sign detection, they all have their own advantages and disadvantages.

RETRACTED

### 2.2. Research Status of Traffic Sign Recognition

Traffic sign recognition is the final goal of the whole detection and recognition process after detection. The commonly used methods include template matching method, neural network classification method, syntax classification method, and so on. Template matching method is a kind of traffic sign recognition algorithm designed for static images, which is widely used. Piccioli et al. [26] used standard traffic signs as shape templates to propose a recognition method based on template matching. The matching degree is obtained by mutual calculation between the set threshold and the input image. This method can better resist different light intensities. There are many reasons for inaccurate matching in the actual matching process. The most common is that the image to be matched may be deformed or blocked, which is quite different from the standard template. In order to reduce the impact of image deformation on the performance of the algorithm, the algorithm [10] performs distance transformation on the input image, which improves the robustness of the algorithm to deformation to a certain extent.

Statistical pattern recognition is also a commonly used classification and recognition method, which has formed a complete theoretical system. Through feature extraction and feature selection, make full use of all kinds of distribution features to divide the region into the feature space, and then combine with the classifier to classify. Xie et al. have achieved high accuracy by extracting hog features from grayscale images and cooperating with SVM for classification [39]. When extracting features, we can use some rotation and scale invariant features, such as the well-known SIFT features with translation and rotation invariance, and PCA features. Fleyeh first zooms the image to a fixed size, uses PCA to extract the feature vector value, and forms a feature vector input classifier, which has a high accuracy. However, two points should be paid attention to when using this algorithm. First, PCA is highly sensitive to rotation, so it is necessary to register the input image when using this algorithm. Second, the adaptability to occlusion is not strong. If there is an occluded part of the logo, the recognition rate will be greatly reduced.

Neural network classification algorithm is a common classifier. It is proposed based on the abstraction of human brain neural network from the perspective of information processing, so as to establish a simple model. Different connection modes can form different networks. The focus is to construct threshold logic units. Neural network has made breakthroughs in many fields. It has the functions of self-organization, self-learning, and association. It is a nonlinear model with good robustness and fault tolerance. Common artificial neural networks include three-layer BP neural network, Hopfield neural network algorithm, etc. In order to achieve the final classification, all pixels of the regularized traffic sign image can be used as feature input. Some researchers use Hu moment invariants of traffic sign images as features and BP neural network as classifier to select the number of nodes of hidden layer according to experience. Neural network usually has a large number of training sets and slow convergence speed. The optimized hidden layer and parameters are uncertain, so it is necessary to adjust the parameters through repeated experiments. In recent years, many scholars have done a lot of research on the input of neural network. Some have extracted the SIFT features of images as input, combined with multi-layer neural network classifiers for classification, and achieved good recognition results [16]. However, this requires high-quality images to be mentioned. If the resolution of the input images is low, the accuracy of SIFT feature extraction will decline; experiments show that wavelet transform can reduce the complexity of the background and resist deformation. The researchers first use Gabor wavelet transform and then use neural network classifier to identify traffic signs. The final results not only improve the classification accuracy, but also greatly speed up the processing speed. AdaBoost improves the classification performance by training multiple classifiers with different parameters and combining the classification results of each classifier. This is a typical ensemble learning classification algorithm. Paclik et al. combined with the characteristics of the color and shape of traffic signs, used the decision tree to divide the signs into several categories, extracted some features of the classified images according to the global nature of the images, used the Laplace classifier for classification, and also obtained good classification results.

RETRACTED

When the object becomes complex, the numerical features cannot fully reflect the information of the image, so it is impossible to fully describe the image features only by extracting the numerical features of the image. At this time, syntactic classification began to enter the attention center of researchers. However, syntactic classification still has many deficiencies in knowledge representation and analysis, which need to be further improved. Almost all of the above detection and identification algorithms detect and identify on their own unpublished data sets, so it is impossible to directly compare the performance of the algorithms. In view of this, the international neural network joint conference IJCNN held a traffic sign classification competition called German traffic sign recognition benchmark (GTSRB) in 2011 and then announced the data set and provided free download service. In 2013, a traffic sign detection competition was held, in which the GTSDB data set was published. The above data sets are collected in the natural traffic environment, which truly simulates various adverse factors such as illumination, tilt, and occlusion that may be affected by the pictures taken during the driving of the car and ensuring the adequacy of the samples, and can comprehensively show the performance of the algorithm.

## 3. Identification of Traffic Signs

The research content of this paper is traffic sign recognition based on optimized convolutional neural network. The traffic sign outside the vehicle is obtained through the camera on the vehicle, and the obtained traffic sign image is input into the computer. The computer completes the detection and recognition of traffic signs after systematic analysis. Because all traffic signs are exposed to natural scenes, and it is also a dynamic target recognition problem, it can deal with more complex adverse situations than in static natural scenes. As can be seen from Figure 1, the identification algorithm flow of traffic signs includes partial preprocessing, feature extraction, classification, and other steps for the regions of interest obtained from the detection process.

Because traffic signs have obvious color and shape features, this paper uses a traffic sign detection method based on color and shape matching to extract Rios, so that it can be more accurate in the next recognition process. The extraction process of Rios has three steps: color conversion; shape matching; and refining Rios. The improved color conversion method is used. After the trained SVM is converted to the gray image, the Rios are found based on the shape template matching. The purpose is to find and retain the regions of interest that are more likely to contain traffic signs. It only needs to be further refined on the Rios obtained on the basis of the first two parts. Input the obtained Rios into Yolo convolutional neural network to detect whether there are Rios.

### 3.1. Image Preprocessing

Preprocessing is to eliminate noise (mainly based on defogging), restore the image with good color intensity and definition, and input it to the subsequent process. However, Rios are vulnerable to a variety of environmental interference, which affects the final classification results. Therefore, before the recognition process, the image preprocessing is used to improve the classification results. Specifically, for the Rios area in the GTSRB data set, there may be 10% of the edge areas around each traffic sign. These edge areas belong to useless areas, which increase the computational complexity. In addition, the traffic signs may not be in the middle of the picture. Therefore, the first thing we need to do is to remove the edge area around the traffic signs. The size of the whole Rios is different, and it is not square. In order to meet the requirements of convolutional neural network, the image with edges removed is uniformly scaled into a square. In this algorithm, it is 48 × 48. Because the contrast value between the image and the image is inconsistent, the image needs to be further normalized. Three contrast normalization methods, image adjustment, histogram equalization, and restricted contrast histogram, are adopted.

RETRACTED

At the same time, in order to make the processing steps more contrast the corresponding grayscale images were used for comparison, and a total of 8 different data sets were used for comparison experiments. The first line to the fourth line from the left are the original image, the image after image adjustment, the image after histogram equalization, and the image after CLAHE method. Each line on the right has a corresponding gray image on the left, and the pixel size is 48 × 48. In view of the characteristics of the traffic signs in this paper, it is necessary to retain the characteristics of the original data set as much as possible. Therefore, ZCA whitening operation is adopted in the image whitening operation in this paper. The preprocessing stage of this image is completed, and the flowchart is shown in Figure 2.

### 3.2. Yolo Classification Model for Traffic Sign Recognition

In order to solve the existing challenges, this paper proposes a Yolo classification model for traffic sign recognition. The proposed model is based on the classical architecture of Yolo (as shown in Figure 3) and applied to traffic sign recognition. The model is a convolutional neural network model, including convolutional and pooling operations.

The convolutional layer applies a discrete convolutional form between the input tensor (e.g., images with different channels) and the small two-dimensional array *f* called filter or convolutional kernel. The mathematical expression of the discrete two-dimensional convolutional process between *F* and *G* is shown in

(1) $$\begin{array}{c} \left(f*g\right)\left(x,y\right)=\sum_{i=-\infty }^{\infty }\sum_{j=-\infty }^{\infty }g\left(i,j\right)f\left(x-i,y-j\right), \end{array}$$

where *x* and *y* are two variables of *F* and *G*, such as rows and columns of pixels, and *I* and *j* are index values that move *f* to *g*. Each layer contains a set of filters, and each filter is responsible for a certain area of the input part.

RETRACTED

The pooling layer, also known as the sub-sampling layer, aims to reduce the spatial resolution of the input and remove redundant information. The pooling layer is composed of an empty core with step value. The most popular pooling methods are maximum pooling and average pooling. Maximum pooling is mainly to extract the highest value perceived by the kernel, and average pooling is mainly to obtain the arithmetic mean value perceived by the kernel.

## 4. Experiment

### 4.1. Experimental Data Set

GTSDB data set is the data set published in the 2013 IJCNN competition. It is a static picture detection data set. All images in the data set are collected from the real traffic environment in different scenes in Germany. The data set was officially released after the competition and later used as a unified standard data set for traffic identification algorithm. The data set was collected for nearly 10 hours, and the video was taken by camera when driving in different streets in Germany during the day. It includes 43 types of traffic signs. The whole data set includes 51839 images in total, and the training set and test set are 39209 and 12630, respectively. The proportion of each type of sample in the data set is different. There is only one traffic sign in each picture, and it is located in the central part of the picture, which is equivalent to Rios as a whole. There are usually some edges around each traffic sign. Because the traffic signs are obtained by shooting video in a moving vehicle, the size of the traffic signs obtained is different due to the inconsistent environment and angle when shooting. There are also pictures affected by light intensity, occlusion, and low resolution, as well as blurring caused by motion. To sum up, these data are a good simulation in the actual scene and can well predict the performance of the algorithm.

### 4.2. Experimental Results and Analysis

The algorithm is tested in detail on GTSRB data set. The optimized convolutional neural network is used to identify 43 traffic categories in the data. The network needs to be trained first with the training set. The training set of GTSRB includes 39209 images. There are 12630 pieces in the test set. GTSRB data set can be divided into several categories according to the unique characteristics and properties of various signs: speed limit signs, other prohibition signs, lifting prohibition signs, indication signs, warning signs, and other signs. The reason for this division is that the first five types of signs have their own unique color and shape characteristics. Other signs actually contain four types of signs, but the similarity of these four types of features is not obvious, which is different from the first five categories. Therefore, they are unified into the sixth category. The algorithm flow of rough classification is relatively simple. First, it is processed according to the above preprocessing steps and then input to the optimized convolutional neural network to extract features and carry out large-scale classification. The first is the training process. The whole data set is batched, and each batch contains a certain amount of data. In this experiment, 100 pictures are input into the training network each time, and the amount of data contained in each batch here is 100. This training method is called batch training, which is commonly used in the training of neural networks. Then, the forward propagation process obtains the error rate, which is also the error rate of this batch of images, and then uses the error to derive the weight and offset according to the back propagation to update these learning parameters.

RETRACTED

It can be seen from Table 1 that the classification accuracy of rough classification has reached more than 95%, which is generally high. In the 12630 samples of the test set, only 136 identifications were incorrectly identified, and the total accuracy rate reached 98.93%. The main reason is that the proposed network can effectively resist image position transformation, scaling, and other forms of distortion.

For the subclassification of traffic signs, since the rough classification has distinguished the major categories to which different traffic signs belong, the subclassification algorithm needs to determine which traffic sign is based on the characteristics of different categories. In the first step, in order to eliminate the influence of edges and other aspects on the identification preprocessing, the optimized convolutional neural network after processing is used to identify the final classification results. Generally, the network parameters trained with the wrong data sets will have large deviation, which is not as good as the actual fitting. Therefore, if the result of rough classification is directly input into the network, the final result is not ideal. This is because the coarse classification results contain misclassification images, which can be used to train the fine classification network so that the fine classification results are not accurate. In order to make the convolutional neural network optimized in the subdivision stage better fit the training data, we set up the network training independence of coarse classification and fine classification, that is, use the original data to train the network.

RETRACTED

Since rough classification has classified several categories, each category provides a corresponding class label. In the subdivision class stage, the traffic sign images belonging to the same class label are used as a sub-data set as input to train the network and classifier. Similarly, preprocessing is carried out according to the characteristics of different class labels. As in the coarse classification stage, the input image size is 48 × 48.

#### 4.2.1. Subclassification of Speed Limit Signs

The speed limit sign contains 8 categories. According to its characteristics, we first split it and reduce it to 48 × 48 pixels, and keep the key part of the logo as much as possible. The output categories designed by the classifier are 8. The specific training test and the structure of the network are similar to those in the rough classification stage. The classification accuracy achieved in the test set is 98.58%.

#### 4.2.2. Subclassification of Identification

The characteristics of the indication signs have been described above. The outer borders of the data set are circular, the background is blue, and the middle is inlaid with indication arrows in different directions. The shape or direction of the indication arrows varies according to the road traffic demand. Therefore, this point can be used as a division to distinguish the indication marks. Before subdividing the class, it does not need to be segmented. It is directly input to the optimized convolutional neural network to extract features and classify. The classifier output indicating the identification is designed as 8 according to the category output. Finally, on the test set, the correct rate of the subdivision class of the indicator is 97.91%.

#### 4.2.3. Subclassification of Warning Signs

The characteristics of warning signs are prominent. Except that the key areas of warning signs such as signal lamps are color patterns, the key areas of other warning signs are basically black and white, and the types of patterns are also very different. Therefore, the key region image is first transformed into gray image and then processed according to the contrast enhancement introduced in the preprocessing, so as to improve the ability of distinguishing between feature classes. Finally, input to the network for classification. There are 15 categories of warning signs in the data set, and 15 classifiers are designed. The accuracy of subclassification on the test set is 98.21%.

RETRACTED

#### 4.2.4. Subclassification of Other Signs

Other signs here include other prohibitions, lifting prohibitions, and other three categories of signs. Because the differences between classes are large, there is no need to partition the identification of the three classes, and the three classes have the same classification network structure. Whether it is the lifting of prohibition, other prohibitions, or others, there are four kinds of identifications. Therefore, in the output design of the classifier, these three identifications are designed as four outputs. On the GTSRB test set, the accuracy of subclassification is 93.33% for lifting the ban, 97.41% for other bans, and 97.99% for others.

### 4.3. Comparison and Analysis with Baseline

Based on the above experimental results, it is concluded that the hierarchical classification algorithm proposed in this paper for the characteristics of traffic signs classifies the test set data on the GTSRB data set with a total accuracy of 98.58%, and the total number of recognition errors is 249. The specific statistics of the number of recognition errors in each category are shown in Table 2. Here, the cause analysis of the error identification may be as follows: partial occlusion is too serious, the scoring rate is too low, motion causes blur, etc.

In order to illustrate the performance of the algorithm proposed in this chapter, the accuracy of the algorithm is compared with that of the international mainstream algorithm, as shown in Table 3. It includes the classification algorithms MCDNN (multi-column depth neural network) and MSCNN (multi-scale convolutional neural network) that have all used convolutional neural networks, and the random forest and LDA methods that have all used hog features. The algorithm in this paper is better than random forest and LDA, and the classification result is roughly the same as that of human performance, but there is still a gap compared with the best result in traffic sign recognition.

In terms of the time complexity of the algorithm, the MCDNN algorithm that achieves the best effect on the GTSRB data set has a training time of 37 hours, and it also takes several hours to test the identification classification on the test set. However, the training time of this algorithm on MATLAB 2015a is about 8 hours, and the test time on the test set is about 40 minutes. The comprehensive results show that the time complexity of this algorithm is much lower than that of similar algorithms, and it meets the requirements of high real time in the proposed application environment.

## 5. Conclusion

Road traffic signs play an important role in transmitting road information and avoiding traffic accidents. And with the development of intelligent transportation, people's awareness of traffic safety is getting higher and higher. With the development of technology, the research on traffic sign recognition has been booming at home and abroad. The actual problem is that our environment is complex and changeable, and traffic signs are likely to be affected by many adverse factors, such as weather, local occlusion, and motion blur. And the identification of road traffic signs is carried out in an environment with high real-time requirements. In this paper, the application of convolutional neural network in traffic sign detection and classification is deeply studied. Traffic sign detection and recognition is a real scene research, which cannot avoid the actual impact of various adverse environmental factors, which increases the difficulty of recognition, and is more challenging than the traffic sign detection technology in static pictures. Therefore, in the future research, the recognition system will be more mature and can combine more technologies. For example, in the aspect of traffic sign detection and recognition algorithm, feature extraction can be combined with visual behavior model. Based on the bionic algorithm, the model vividly simulates the process of biological image and increases the recognition accuracy.

RETRACTED

## Figures and Tables

**Figure 1:** Identification algorithm flow of traffic signs.

**Figure 2:** Whole process of image processing.

**Figure 3:** Yolo model.

**Table 1:** Results of rough classification.

	Number of classification errors	Probability (%)
Speed limit sign	31	98.97
Other prohibition signs	14	97.76
Lifting prohibition sign	15	96.78
Indication mark	17	98.56
Warning sign	32	98.77
Other identification	28	98.54

**Table 2:** Number of error identification marks of each category.

	Speed limit	Other prohibitions	Lifting the ban	Warning	Indicate	Other
个数	59	38	24	50	37	41

**Table 3:** Comparison of recognition results between this algorithm and other algorithms.

	Speed limit	Other prohibitions	Lifting the ban	Indicate	Warning	Other	Total
MCDNN	99.52	98.93	99.78	99.91	98.98	99.31	99.55
MSCNN	98.71	99.85	94.44	97.23	98.14	98.81	98.26
RF	95.97	99.15	86.49	98.97	92.11	98.81	96.23
Human performance	97.63	99.93	98.89	99.72	99.72	98.67	98.84
LDA	95.37	96.80	85.83	97.18	93.73	98.73	95.68
Our	98.61	97.41	93.33	97.91	98.21	97.99	98.37

## Data Availability

The data set can be accessed upon request.
